This article has been retracted.

# Regulation of Chondrocyte Differentiation by miR-455-3p Secreted by Bone Marrow Stem Cells through Phosphatase and Tensin Homolog Deleted on Chromosome Ten/Phosphoinositide 3-Kinase-Protein Kinase B

**DOI:** 10.1155/2023/6738768

**Published:** 2023-02-15

**Authors:** Axiang He, Yaru Liu, Shang Sang, Renbo Zhang, Zheng Jiang, Yanjie Mao, Wanjun Liu

**Affiliations:** ^1^Department of Orthopedics, Shanghai Jiao Tong University Affiliated Sixth People's Hospital, Shanghai 201306, China; ^2^Department of Food Science and Engineering, Shanghai Ocean University, Shanghai 201306, China

## Abstract

The effects of the regulation of phosphatase and tensin homolog deleted on chromosome ten (PTEN) by microribonucleic acid- (miR-) 455-3p on bone marrow stem cells' (BMSCs') chondrogenic development were examined based on the phosphoinositide 3-kinase (PI3K)/protein kinase B (AKT) signal pathway. The alterations in miR-455-3p and PTEN were identified using osteoarthritis (OA) and healthy chondrocytes. Rats raised on the SD diet had their BMSCs isolated for chondrocyte-induced differentiation (blank group), transfected miR-455-3p mimic (mimic group), and inhibitor (inhibitor group). Besides, cell proliferation, alizarin red mineralization staining, and the activity of alkaline phosphatase (ALP) were detected. Real-time fluorescent quantitation polymerase chain reaction (PCR) and Western blot were utilized to detect Runx2, OPN, OSX, COL2A1 mRNA, and the difference between PI3K and AKT. Dual-luciferase reporter (DLR) genes were selected to analyze the target relationship of miR-455-3p to PTEN. It was demonstrated that miR-455-3p in OA was downregulated, while PTEN was upregulated (*P* < 0.05) in comparison to healthy chondrocytes (*P* < 0.05). Versus those in the blank group, alizarin red mineralization staining and the activity of ALP increased; RUNX, OPN, OSX, COL2A1 mRNA, p-PI3K, and p-AKT were elevated in the mimic group (*P* < 0.05). Versus those in the blank and mimic groups, alizarin red mineralization staining and the activity of ALP reduced; RUNX, OPN, OSX, COL2A1 mRNA, p-PI3K, and p-AKT were downregulated in the inhibitor group (*P* < 0.05). miR-455-3p could target PTEN to inhibit its expression, thus activating the PI3K/AKT signal pathway and promoting BMSCs chondrocyte-induced differentiation. The research results provided reference for the occurrence of OA and the study on therapeutic target.

## 1. Introduction

Degenerative osteoarthropathy is also called osteoarthritis (OA), degenerative arthritis, and senile arthritis. The main symptoms of degenerative osteoarthropathy include degenerative injury of articular cartilage (AC) and reactive hyperplasia of joint edge and subchondral bone caused by age, obesity, trauma, and joint deformity [1]. The prevalence of OA has been increasing recently, year over year. Patients' quality of life is significantly impacted by OA-related arthralgia and impairment, which also makes therapy more challenging. The primary pathogenic aspect of OA, along with cartilage matrix degradation and chondrocyte decrease, is the degenerative change in AC. OA frequently occurs in joints with heavy weight and high activity level, such as cervical vertebra, knee joint, and hip joint. The main clinical characteristics of OA include chronic arthralgia, anchylosis, joint swelling, activity limitation, and joint deformity [2]. The OA can be treated by the use of nonsteroidal anti-inflammatory (NSAI) drugs, gene therapy, and surgical therapy. However, side effects of NSAI drugs are very terrible and obvious, surgical therapy is only appropriate for the treatment of end-stage patients, and the clinical application prospect of gene therapy is unclear [3]. Hence, clinical effective treatment method for OA is of great significance for the improvement of quality of life and prognosis for patients.

Because cartilage has a low ability to regenerate, it cannot heal itself after pathological alterations. If it is not addressed in a timely manner, cartilage damage will worsen and eventually result in joint dysfunction [4]. One of the main factors contributing to the worsening of AC damage is the death of many chondrocytes. Osteogenitor stem cells can be formed from bone marrow stem cells (BMSCs). They can build and mend bones by diffusing into chondrocytes or osteoblasts under controlled conditions. BMSCs show self-renewal and the potential for multidirectional differentiation. They can differentiate into osteoblasts, chondroblasts, and adipocytes under the action of cytokines. BMSC transplantation can be used for the treatment of cartilage injury to induce the differentiation of BMSCs into chondrocytes. Besides, it can be applied in the repair of cartilage injury among OA patients. Additionally, BMSCs can undergo directed induction to differentiate into chondrocytes and participate in the rebuilding and repair of cartilaginous tissues. What is more, they can effectively inhibit the apoptosis of chondrocytes and are of importance in repairing cartilage injury for patients with gonitis and OA [5]. Chondrogenic differentiation of BMSCs is affected by micro environment and the levels of multiple cytokines at injured sites. PI3K/AKT is related to cell proliferation, differentiation, and survival. In recent years, it is verified that PI3K/AKT signal pathway can promote the proliferation and differentiation of precursor osteoblasts [6]. Phosphatase and tensin homolog deleted on chromosome ten (PTEN) is the inhibitor of PI3K/AKT signal pathway that can promote the dephosphorylation of PI3K [7]. However, the role of PTEN in BMSC chondrogenic differentiation (CD) is unclear.

An endogenous noncoding RNA molecule (20 nucleotides in length) is known as microRNA (miRNA). By focusing on the 3′ untranslated region of the mRNA, it can restrict mRNA expression as an “absorbent sponge,” which helps to further control the prevalence of illnesses [8]. More and more researches show that miRNA is associated with cartilage and OA. According to Endisha et al. [9], miR-34a-5p was elevated in the cartilages of OA patients, and its suppression helped prevent cartilage injury. It has been demonstrated that miR-455-3p regulates HDAC2 to activate the Nrf2/ARE signal pathway, protect osteoblasts from oxidative stress, and promote osteoblast development [10]. miR-455-3p mimic transfection could promote ALP activity in BMSCs after CD, while miR-455-3p inhibitor transfection inhibits it. Based on above findings, miR-455-3p promotes the CD of BMSCs. PTEN was the target gene of miR-455-3p. At present, the regulation of PTEN by miR-455-3p and its influences on the chondrogenic ability of BMSCs through PI3K/AKT signal pathway were unclear. Hence, the target relationship of miR-455-3p to PTEN was verified. In addition, the effects of miR-455-3p on the proliferation and chondrogenic ability of BMSCs inducing CD and status of PI3K/AKT signal pathway were analyzed. Results in this work provided reference for the occurrence of OA and the study on therapeutic target.

## 2. Materials and Methods

### 2.1. Animals and Reagents

Clean Sprague-Dawley (SD) rats were bought from the Animal Experimental Research Center under the Shanghai Jiao Tong University Affiliated Sixth People's Hospital (SJTU 6# Hospital). Fetal calf serum (FCS), penicillin-streptomycin (PS), Opti-MEM medium, D-MEM/F-12 medium, and FCS were all bought from Gibco Company (USA). Thermo Fisher Scientific Company sold a Lipofectamine 2000 kit and an alkaline phosphatase (ALP) activity detection kit (USA). Methyl thiazolyl tetrazolium (MTT) kit was supplied by Beijing Solarbio Science & Technology Co., Ltd. Osteoblast mineralized nodule staining reagents and Dual-Lumi™ dual-luciferase reporter (DLR) gene kit were from Beyotime Biotechnology Co., Ltd. (Shanghai). PrimeScript™ RT reagent Kit with gDNA Eraser (Perfect Real Time) and TB Green® Premix Ex Taq™ II (Tli RNaseH Plus) kits were from Takara Biomedical Technology (Beijing) Co., Ltd. GAPDH, PTEN, PI3K, p-PI3K, AKT, p-AKT first antibodies, and horseradish peroxidase- (HRP-) labeled IgG second antibody were purchased from Abcam Company (UK).

### 2.2. Experimental Methods

#### 2.2.1. Segregation and Culture of Chondrocytes

Five patients with abandoned cartilage tissues undergoing total hip replacement for femoral fracture caused by trauma at the SJTU 6# Hospital were selected, including 3 males and 2 females in 35.26 ± 1.93 years old. Besides, 5 OA patients with abandoned cartilage tissues undergoing total hip replacement were selected, including 2 males and 3 females in 62.19 ± 4.05 years old. The research had been approved by Medical Ethics Committee under the SJTU 6# Hospital, and all patients had signed informed consent forms. First, the acquired cartilage tissues were rinsed with physiological saline carefully. After being cut into small pieces with the volume of 1 mm^3^, they were added with 5 mg/mL protease digested tissue for 1.5 h and 0.25 mg/mL collagenase P digested tissue for 6 h. Next, they were centrifuged at 1,000 rpm for 10 min to collect the cell precipitation, which was supplemented with D-MEM/F-12 cell culture medium containing 10% FCS and 1% PS. After being shaken evenly, it was incubated with 5% CO_2_ at 37°C for routine cell culture.

#### 2.2.2. Segregation, Culture, and Identification of BMSCs

10 healthy male SD rats aged about 1 month were selected. Their average weight was 104.55 ± 8.63 g. The implementation of the research had been approved by Animal Experiment Ethics Committee under SJTU 6# Hospital. The experimental protocols complied with national laws. Bilateral femurs were removed to reveal the bone medullary chamber in sterile condition after the rats were killed using the cervical dislocation method. The bone marrow was then flushed out of bone medullary cavity using necessary volume of D-MEM/F-12 medium, which was extracted using a 2 mL syringe. BMSCs were then divided and cultivated using the adherent segregation method. During the transfer of culture of the 3rd generation, BMSCs were digested, centrifuged, and resuspended. Next, they underwent inoculation in a 96-well plate after concentration was adjusted to 1 × 10^9^/L. Then, they were added with CD34, CD44, CD45, and CD90 antibodies and incubated away from light at normal temperature for half an hour. After PBS washing, the cells were resuspended. Finally, the positive rate of surface antibodies was detected with a flow cytometer (FCM).

#### 2.2.3. Induction of CD

BMSCs cultured in the 4th passage were performed with induction of CD. When 80% cells were fused, they were digested with 0.25% trypsin. After being centrifuged, the cells underwent counting and then were inoculated into a 12-well plate at 1.5 × 10^5^/cm^2^ and routinely cultured for 24 hours. At this time, routine medium was replaced with chondrogenic induction medium (10% FCS, 1% PS, 0.1 *μ*M dexamethasone, 10 mmoL/L *β*-glycerophosphoric acid, 50 *μ*moL/L vitamin C, and D-MEM/F-12 culture medium were contained). After that, the cells were routinely cultured, and the medium was updated every 3 days.

#### 2.2.4. Cell Transfection and Grouping

Normal BMSCs were acquired and enrolled in the control group (Ctrl), and BMSCs induced by CD were rolled into a blank group (blank), a negative control group (NC), a miR-455-3p mimic group (mimic group), and a miR-455-3p inhibitor group (inhibitor group). The normal BMSCs were inoculated into the 96-well plate at 5 × 10^4^/well. When cell confluence amounted to about 50%, Lipofectamine 2,000 transfection experiment was performed. Besides, Opti-MEM medium was utilized to dilute reagent Lipo2000, miR-455-3p mimic and inhibitor, and NC. After being mixed evenly, it was stood by for 5 minutes. Next, it was mixed with Lipo2000+ NC, Lipo2000 + miR-455-3p mimic, and Lipo2000 + miR-455-3p inhibitor, respectively. Then, it was stood for 20 minutes after being mixed evenly. After finishing above operations, the original medium was discarded and the Opti-MEM medium was adopted newly. Then, it was added with mixture and cultured. After 6 hours, Opti-MEM medium was cleared and the routine medium was added for further culture.

#### 2.2.5. Detection of Cell Proliferation

The 96-well plate was filled with the cells, which were then clustered. At 6 h, 12 h, 24 h, 48 h, and 72 h after the culture, in each well, 20 L of 5 mg/mL MTT reagent was employed. Then, cells were put in the incubator at 37°C for 4 hours. Supernatant was eliminated and 100 *μ*L dimethyl sulfoxide (DMSO). Next, the cells were oscillated and incubated on a constant-temperature shaking table for 20 minutes. Blank was set as the control group. The absorbance (optical density (OD)) of each well was detected at 490 nm with a multifunctional microplate reader. Finally, the proliferative activity of cells was detected based on the equation (OD_purpose_/OD_control_ − 1) × 100%.

#### 2.2.6. Alizarin Red Mineralization Staining and Quantitative Detection

The processed cells were extracted and rinsed with PBS. After that, they were soaked in 4% polyformaldehyde (POM) for fixation for around 30 minutes, washed with PBS, and added with 1% alizarin red (pH = 4.3) staining solution. Next, they were incubated naturally for about 20 minutes. After that, floating color was rinsed with PBS, and then, 1 mL PBS was added into the cells. Mineralized nodule staining in the cells was observed using an inverted microscope. After photo-taking, mineralized nodules were extracted with 10% cetylpyridinium chloride (CPC). Besides, 200 *μ*L solution was absorbed and then placed in the 96-well plate. Finally, the multifunctional microplate reader was employed for the detection of OD values at the wavelength of 562 nm.

#### 2.2.7. Detection of ALP Activity

The processed cells were extracted and then added with RIPA solution for cytolysis. After lysis buffer was collected, the cells were centrifuged at 12,000 rpm and 4°C, and this process should last for 20 minutes so that the supernatant could be fully extracted and placed in the reaction hole. At 37°C, the cells were incubated at a constant temperature. After that, the reaction should be terminated. A multifunctional microplate reader was employed to detect OD value at 405 nm. In addition, quinaldic acid (BCA) kit was utilized to detect protein concentration. The absorbance of per gram of protein reacting for 15 minutes was defined as ALP activity.

#### 2.2.8. Real-Time Fluorescent Quantitation Polymerase Chain Reaction (PCR) Detection

The processed cells were extracted, and total RNA was extracted according to TRIzol method. Besides, the concentration and mass of RNA were extracted. After an appropriate amount of RNA was extracted, cDNA was reversely transcribed according to the instruction of 1st-strand cDNA synthesis kit. cDNA was used as the template for the preparation of 10 *μ*L real-time fluorescent quantitation PCR reaction system. cDNA, SYBR Premix EX Taq™, upstream and downstream primers, and ddH_2_O were added. The reaction environment was defined as 95°C for 30 s, 95°C for 5 s, 60°C for 35 s (40 cycles), and 72°C for 3 min. The sequence of quantitation primers of target genes was GAPDH (F) 5′-ATGGGACGATGCTGGTACTGA-3′, (R) 5′-TGCTGACAACCTTGAGTGAAAT-3′; Runx2 (F) 5′-TTCAACGATCTGAGATTTGTGGG-3′, (R) 5′-GGATGAGGAATGCGCCCTA-3′; OPN (F) 5′-AGCAAGAAACTCTTCCAAGCAA-3′, (R) 5′-GTGAGATTCGTCAGATTCATCCG-3′; OSX (F) 5′-ACCCCAAGATGTCTATAAGCCC-3′, (R) 5′-CGCTCTAGCTCCTGACAGTTG-3′; COL2A1 (F) 5′-CAGGATGCCCGAAAATTAGGG-3′, (R) 5′-ACCACGATCACCTCTGGGT-3′; and PTEN (F) 5′-TTCTTCCGCCAGTCGGTAG-3′, (R) 5′-CTGCTTCTCCTCGATCAGCC-3′. GAPDH was set as the internal reference gene. Expression of target genes was detected according to 2^-△△Ct^.

#### 2.2.9. Western Blot Detection

The processed cells were extracted and added with RIPA solution for cytolysis to extract total protein. According to the instructions of BCA kit, the concentration of extracted proteins was quantitatively detected. Then, an appropriate amount of proteins was extracted and added with loading buffer. Next, they were mixed evenly and heated for denaturation. The proteins were segregated by preparing polyacrylamide gel electrophoresis (PAGE) with the concentration consistent with the amount of protein molecules. After PAGE was loaded, the target genes were transferred onto polyvinylidenefluoride (PVDF) membrane, which was then sealed with blocking solution containing 5% skim milk powder. Next, it was added with diluted GAPDH, PTEN, PI3K, p-PI3K, AKT, and p-AKT first antibodies (1 : 2000) and then incubated at 4°C for the whole night. After being cleaned with TBST, the PVDF membrane was added with HRP-labeled IgG second antibody (1 : 3000) and then incubated for 1 h. Again, after TBST washing, enhanced chemiluminescence (ECL) detection kit was employed for development and then placed into the gel imager for imaging and photo-taking. Finally, ImageJ software was adopted for the quantitation detection of relative grayscale values of protein bands.

#### 2.2.10. DLR Gene Detection

The binding target of PTEN and miR-455-3p was predicted using miRBase and TargetScan. The information about 3′-UTR of PCR amplified wild-type (WT) PTEN and mutant (MUT) PTEN genes and PCR amplified primer of WT-PTENd included (F) 5′-GATCGCTCGAGTTTCAATCATAATACCTGC-3′ and (R) 5′-GCGGCCAGCGGCCGCT TCTGCCAAATACTACAGTTA-3′. The information about PCR amplified primer of MUT-PTENd included (F) 5′-TTTGTGAGCCCCTCCTTCCCACCGGAAGTC-3′ and (R) 5′-GGACTTCCGGTGGGAAGGAGGGCTCACAAAC-3′. The amplified gene sequence was ligated with pcDNA-3.1(+) vector to construct the expression vectors of WT- and MUT-PTEN genes. After that, WT-PTEN and MUT-PTEN were transfected into 293T cells in miR-455-3p NC and miR-455-3p mimic. In addition, DLR gene kit was employed to detect the activity of firefly luciferase and Renilla luciferase.

### 2.3. Statistical Analysis

SPSS 19.0 was employed for data statistical analysis of experimental data. All experimental data were denoted by mean ± standard deviation ($\bar{x}\pm s$). The independent sample *t*-test and ANOVA were used to compare the two groups and multiple groups, respectively. *P* < 0.05 suggested that the difference was statistically significant.

## 3. Results

### 3.1. Differences in miR-455-3p and PTEN Expressions in OA and Healthy Cartilages

The differences in miR-455-3p and PTEN in chondrocytes between OA patients and healthy people were compared. Versus that in healthy chondrocytes, miR-455-3p expression apparently decreased (Figure 1(a)) while PTEN notably improved (Figure 1(b)) in chondrocytes among OA patients.

### 3.2. Verification of the Effects of Overexpressed/Silencing miR-455-3p

The differences in miR-455-3p and PTEN expressions in BMSCs among all groups were investigated. According to the detection of miR-455-3p (Figure 2(a)), miR-455-3p was upregulated in the blank, NC, and mimic groups in contrast to that in the Ctrl group. miR-455-3p was decreased in the inhibitor group (*P* < 0.05). miR-455-3p in blank exhibited no observable difference with that in the NC group (*P* > 0.05). Versus that in the blank and NC groups, miR-455-3p in the mimic group was upregulated, and that in the inhibitor group was downregulated (*P* < 0.05). According to the detection of PTEN expression (Figure 2(b)), PTEN expression in cells in the blank, NC, and mimic groups was downregulated, while that in the inhibitor group was elevated in contrast to that in the Ctrl group (*P* < 0.05). No remarkable change was detected in PTEN in the blank and NC groups (*P* > 0.05). In contrast to that in the blank and NC groups, PTEN in the mimic group was downregulated, while that was upregulated in the inhibitor group (*P* < 0.05).

### 3.3. Influences of miR-455-3p Expression on BMSC Proliferation

It was discovered that there were variations in each group's BMSC proliferative activity. Proliferative activity of BMSCs gradually increased in all groups as the culture developed. The mimic group had the maximum proliferative activity, whereas the inhibitor group had the lowest proliferative activity. Proliferative activity of BMSCs increased in other three groups compared to the Ctrl and inhibitor groups (*P* < 0.05). Versus that in the blank and NC groups, proliferative activity of the mimic group increased, while that in the inhibitor group reduced (*P* < 0.05). All the above descriptions could be checked in Figure 3.

### 3.4. Influences of miR-455-3p on Alizarin Red Mineralization Staining in BMSCs

In all groups, variations in the alizarin red mineralization staining of BMSCs were found. The mimic group had the biggest area of alizarin red mineralization staining, which was followed by the blank and NC groups. Following alizarin red mineralization staining, cell absorbance was determined. Versus that in the Ctrl group, cell absorbance in the blank, NC, and mimic groups was improved after alizarin red mineralization staining (*P* < 0.05). Great difference was not detected in cell absorbance in the blank and NC groups after alizarin red mineralization staining (*P* > 0.05), based on which the cell absorbance in the mimic group was enhanced after alizarin red mineralization staining, while that in the inhibitor group decreased after alizarin red mineralization staining (*P* < 0.05).  Figure 4 illustrates the specific influences of miR-455-3p on alizarin red mineralization staining in BMSCs.

### 3.5. Influences of miR-455-3p on ALP Activity in BMSCs

Figure 5 exhibits the influence of miR-455-3p on ALP activity in BMSCs, which showed that there were variations in the ALP activity of BMSCs across the groups. ALP stained bluish violet in BMSCs. The mimic group had the most positive stained ALP results, followed by the blank and NC groups (Figure 5(a)). ALP activity was calculated (Figure 5(b)). Versus that in the Ctrl group, ALP activity in the blank, NC, and mimic groups increased (*P* < 0.05). Remarkable difference was hard to be detected in ALP activity from the blank and NC groups (*P* > 0.05), based on which the ALP activity was enhanced in the mimic group and was reduced in the inhibitor group (*P* < 0.05).

### 3.6. Influences of miR-455-3p on ALP Activity in Ability of CD in BMSCs

Influences of miR-455-3p on ALP activity in ability of CD in BMSCs are given in Figure 6. It could be observed that the expression differences of Runx2, OPN, OSX, and COL2A1 mRNA in BMSCs of all groups were detected by real-time fluorescent quantitation PCR (Figures 6(a)–6(d)). Versus those in the Ctrl group, Runx2, OPN, OSX, and COL2A1 mRNA in the blank, NC, and mimic groups were upregulated (*P* < 0.05). No remarkable difference was detected in Runx2, OPN, OSX, and COL2A1 mRNA between the blank and NC groups (*P* > 0.05). Based on the blank and NC groups, the Runx2, OPN, OSX, and COL2A1 mRNA in the mimic group were upregulated, while those in the inhibitor group were downregulated (*P* < 0.05). Besides, no apparent difference was detected in Runx2, OPN, OSX, and COL2A1 mRNA between the Ctrl and Inhibitor groups (*P* > 0.05).

### 3.7. Influences of miR-455-3p on PI3K/AKT Signal Pathway in BMSCs

PI3K/AKT is related to cell proliferation, differentiation, and survival. In recent years, it is verified that PI3K/AKT signal pathway can promote the proliferation and differentiation of precursor osteoblasts. The PTEN and PI3K/AKT signal pathway protein expressions in BMSCs from all groups were detected, as given in Figures 7(a)–7(d). Among them, Figures 7(a)–7(d) show the Western blot graph, expression of PTEN, phosphorylation level of p-PI3K, and phosphorylation level of p-AKT, respectively. PTEN expression was downregulated compared to those in the Ctrl group, while p-PI3K and p-AKT were upregulated in the blank, NC, and mimic groups (*P* < 0.05). Versus those in the Ctrl group, PTEN was upregulated in the inhibitor group (*P* < 0.05). They showed no visible difference between the blank and NC groups (*P* > 0.05). Versus those in the blank and NC groups, PTEN was downregulated, while p-PI3K and p-AKT were elevated in the mimic group (*P* < 0.05). Versus the blank and NC groups, PTEN was elevated, while p-PI3K and p-AKT were downregulated in the inhibitor group (*P* < 0.05).

### 3.8. Verification of Target Relationship of miR-455-3p to PTEN

Firstly, the target binding position in 3′UTR of miR-455-3p and PTEN was predicted. It was found that there were the complementary pairings of 7 bases (Figure 8(a)). Next, the influences of the cotransfection of WT-PTEN and MUT-PTEN with miR-455-3p on luciferase activity ratio were verified, as illustrated in Figure 8(b). It was demonstrated that DLR activity ratio apparently increased after the cotransfection of WT-PTEN and MUT-PTEN with miR-455-3p (*P* < 0.05).

## 4. Discussion

The prevalence of OA has been increasing recently, year over year. Patients' quality of life is significantly impacted by OA-related arthralgia and impairment, which also makes therapy more challenging [11]. The primary pathogenic aspect of OA, along with cartilage matrix degradation and chondrocyte decrease, is the degenerative change in AC. OA frequently occurs in joints with heavy weight and high activity level, such as cervical vertebra, knee joint, and hip joint. The main clinical characteristics of OA include chronic arthralgia, anchylosis, joint swelling, activity limitation, and joint deformity. BMSCs have the capacity for self-renewal and the potential for multidirectional differentiation. They can differentiate into osteoblasts, chondroblasts, and adipocytes under the action of cytokines [12]. BMSC transplantation can be used for the treatment of cartilage injury to induce the differentiation of BMSCs into chondrocytes. Besides, it can be applied in the repair of cartilage injury among OA patients [13]. Hence, clinical effective treatment method for OA is of great significance for the improvement of quality of life and prognosis for patients.

miR-455-3p is proved to involve in the onset and progression of numerous disorders, including cancer, pulmonary fibrosis, and OA [14–16]. In the study, miR-455-3p varied between cartilaginous tissues with OA and those that were in good health. It was found that in cartilaginous tissues of OA patients, miR-455-3p was elevated and PTEN showed the opposite case. Therefore, it was hypothesised that PTEN and miR-455-3p were implicated in the development and ageing of cartilages in OA. Additionally, miR-455-3p inhibitor and mimic were transfected, and the effects on BMSC proliferation brought on by CD were examined. It was found that miR-455-3p mimic was conductive to proliferation of BMSCs after transfection. After CD, alizarin red mineralization staining was analyzed. After the transfection of miR-455-3p mimic, more BMSCs were mineralized. ALP was widely distributed in the liver, kidney, and small intestine and usually viewed as the assessment indicator for osteogenesis [17, 18]. According to the research results, miR-455-3p mimic transfection could promote ALP activity in BMSCs after CD, while miR-455-3p inhibitor transfection inhibits it. Based on above findings, miR-455-3p promotes the CD of BMSCs.

Runx2 can induce and promote the maturation of osteocyte and the differentiation of osteoblasts. Some studies confirm that the inhibition of Runx2 can slow down the progression of OA and further gets involved in OA [19]. OPN refers to osteopontin, which is glycosylated protein and an important bone matrix protein. It is closely associated with osteogenesis and its occurrence [20]. Osterix (OSX) is a type of specific transcription factor of osteoblasts, which is indispensable in the process of osteogenesis [21]. COL2A1 mainly encodes and synthesizes type II collagen, which is involved in ossification in periosteum and endochondral ossification. It is reported that COL2A1 mutation leads to various skeleton-cartilage dysplasia diseases [22, 23]. In the research, influences of miR-455-3p on Runx2, OPN, OSX, and COL2A1 expressions were investigated. It was suggested that Runx2, OPN, OSX, and COL2A1 were upregulated in BMSCs after miR-455-3p mimic transfection. In contrast, those were downregulated after miR-455-3p inhibitor transfection. miR-455-3p were shown to regulate the CD of BMSCs.

PI3K/AKT signal pathway is involved in various biological processes, such as the occurrence, development, and sequelae of cancer [24]. PI3K/AKT is related to cell proliferation, differentiation, and survival. In recent years, it is verified that PI3K/AKT signal pathway can promote the proliferation and differentiation of precursor osteoblasts. PI3K is a lipid kinase in cytoplasm. After being stimulated and activated by growth factors, it phosphorylates phosphatidylinositol bisphosphate on plasma membrane. AKT refers to serine/threonine kinase. After phosphorylation, it can transmit the signal to mammalian target of rapamycin (mTOR) and effector proteins. In addition, PI3K/AKT gets involved in osteogenic differentiation of BMSCs. Li et al. [25] found that PI3K inhibitor LY294002 inhibited the proliferation of MSCs and further got involved in the healing process of skin wounds. Yu et al. [26] investigated the effect of apolipoprotein D-mediated PI3K/AKT pathway on the osteogenic inhibition of BMSCs. They found that apolipoprotein D reduced glucocorticoid-induced osteogenic inhibition of BMSCs through PI3K/AKT signal pathway and further protected osteoporosis (OP). It was demonstrated that the phosphorylation levels of PI3K and AKT in BMSCs were apparently enhanced after CD, which showed that the activation of PI3K/AKT signal pathway could promote the CD ability of BMSCs. After the transfection of miR-455-3p mimic, the phosphorylation levels of PI3K and AKT in cells were improved more notably. The above results indicated that miR-455-3p could activate PI3K/AKT signal pathway to get involved in the CD of BMSCs.

Being an inhibitor of PI3K/AKT signal pathway, PTEN is involved in the survival, proliferation, and differentiation of tumor cells [27]. It is verified that PTEN participates in occurrence and development of OA [28]. Chen et al. [29] proved that HOTAIR could negatively regulate the expression of target PTEN after miR-20b expression and further get involved in the process of OA. In the research, DLR genes verified that PTEN was the target gene of miR-455-3p. miR-455-3p could target PTEN and downregulate its expression.

## 5. Conclusion

In the cartilage of OA patients, miR-455-3p expression was found to be greatly decreased whereas PTEN expression was elevated. miR-455-3p may target PTEN and subsequently interact with the PI3K/AKT signalling pathway and BMSC development into chondrogenic cells. However, mechanism of miR-455-3p-targeted PTEN in the CD of BMSCs was only verified by cell experiment, which was the shortcoming of this work and should be made up in future. In follow-up research, animal models should be prepared to investigate the repair of cartilage injury among OA patients by miR-455-3p-targeted PTEN. To conclude, the research results provided reference for the occurrence of OA and the study on therapeutic target.

## Figures and Tables

**Figure 1:** Analysis of gene expression profile in OA and healthy cartilages. Note: OA referred to osteoarthritis. (a) miR-455-3p expression. (b) PTEN expression. ^∗^ meant *P* < 0.05.

**Figure 2:** Comparison of expressions of miR-455-3p and PTEN in BMSCs. Note: (a) miR-455-3p. (b) PTEN. A, B, C, and D meant *P* < 0.05 in comparison to the Ctrl, blank, NC, and mimic groups, respectively.

**Figure 3:** Comparison of proliferative activity of BMSCs. Note: A, B, C, and D meant *P* < 0.05 in comparison to the Ctrl, blank, NC, and mimic groups, respectively.

**Figure 4:** Detection of alizarin red mineralization staining in BMSCs. Note: A, B, C, and D meant *P* < 0.05 in comparison to the Ctrl, blank, NC, and mimic groups, respectively.

**Figure 5:** ALP staining and activity detection in BMSCs. (a) Observation on ALP staining in BMSCs (×100). (b) Detection results of ALP activity in BMSCs. Note: A, B, C, and D meant *P* < 0.05 in comparison to the Ctrl, blank, NC, and mimic groups, respectively.

**Figure 6:** Detection of Runx2, OPN, OSX, and COL2A1 mRNA in BMSCs. (a–d) The relative expressions of Runx2, OPN, OSX, and COL2A1 mRNA, respectively. Note: A, B, C, and D meant *P* < 0.05 in comparison to the Ctrl, blank, NC, and mimic groups, respectively.

**Figure 7:** Detections of PTEN, PI3K, and AKT in BMSCs. (a) Western blot graph. (b) Expression of PTEN. (c) Phosphorylation level of p-PI3K. (d) Phosphorylation level of p-AKT. Note: A, B, C, and D meant *P* < 0.05 in comparison to the Ctrl, blank, NC, and mimic groups, respectively.

**Figure 8:** Verification of target binding between miR-455-3p and PTEN. (a) Target binding position. (b). Detection of target relationship by DLR genes. Note: the comparison with WT-PTEN and miR-NC cotransfection group indicated ^∗^*P* < 0.05.

## Data Availability

All data, models, and code generated or used during the study appear in the submitted article.
